# The Prognostic Significance of Different Bleeding Classifications in off-pump coronary artery bypass grafting

**DOI:** 10.1186/s12872-019-01315-0

**Published:** 2020-01-10

**Authors:** Ziwei Xi, Yanan Gao, Zhenxian Yan, Yu-Jie Zhou, Wei Liu

**Affiliations:** Department of Cardiology, Beijing Anzhen hospital, Capital Medical University, Anzhen Road, Chaoyang District, Beijing, 100029 China

**Keywords:** Bleeding, Off-pump coronary artery bypass grafting (OPCAB), European registry of coronary artery bypass grafting (E-CABG), Universal definition of perioperative bleeding (UDPB), Bleeding academic research consortium (BARC)

## Abstract

**Background:**

Perioperative bleeding during cardiac surgery are known to make patients susceptible to adverse outcomes and several bleeding classifications have been developed to stratify the severity of bleeding events. Further validation of different classifications was needed. The aim of present study was to validate and explore the prognostic value of different bleeding classifications in patients undergoing off-pump coronary artery bypass grafting (OPCAB).

**Methods:**

Data on baseline and operative characteristics of 3988 patients who underwent OPCAB in Beijing Anzhen Hospital from February 2008 to December 2014 were available. The primary endpoint was a composite of in-hospital death and nonfatal postoperative myocardial infarction (MI). The secondary endpoint was postoperative acute kidney injury (AKI). We explored the association of major bleeding defined by the European registry of Coronary Artery Bypass Grafting (E-CABG), Universal Definition of Perioperative Bleeding (UDPB), Bleeding Academic Research Consortium (BARC) classification and Study of Platelet Inhibition and Patient Outcomes (PLATO) with primary endpoints by multivariable logistic regression analysis and investigated their significance of adverse event prediction using goodness-of-fit tests of − 2 log likelihood.

**Results:**

In-hospital mortality was 1.23% (*n* = 49) and postoperative MI was observed in 4.76% (*n* = 190) of patients, AKI in 24.69% (*n* = 985). The incidence of the primary outcome was 5.99% (*n* = 239). Multivariable logistic regression analysis showed that BARC type 4 (OR = 2.64, 95% CI: 1.66–4.19, *P* < 0.001), UDPB class 4 (OR = 3.52, 95% CI: 2.05–6.02, P < 0.001) and E-CABG class 2–3 (class 2: OR = 2.24, 95% CI: 1.36–3.70, *P* = 0.001; class 3: OR = 12.65, 95% CI: 2.74–18.43, *P* = 0.002) bleeding but not PLATO bleeding were associated with an increased risk of in-hospital death and postoperative MI. Major bleeding defined by all the four classifications mentioned above was an independent risk factor of AKI after surgery. Inclusion of major bleeding defined by these four classifications improved the predictive performance of the multivariable model with baseline characteristics.

**Conclusions:**

Bleeding assessed by BARC, E-CABG and UDPB classifications were significantly associated with poorer immediate outcomes. These classifications seemed to be valuable tool in the assessment of prognostic effect of perioperative bleeding.

## Background

Perioperative bleeding is a common concern in patients undergoing cardiac surgery [1, 2]. Bleeding complications have been proven to be associated with an increased risk of subsequent adverse outcomes including infection [3], myocardial infarction, stroke, stent thrombosis, and death [4–6].

A variety of definitions of bleeding were proposed to stratify the severity of bleeding which was as an important endpoint to assess the efficacy and safety of procedure [7]. However, different definitions are used across clinical trials and registries, hampering direct comparison across studies [8, 9]. Moreover, few definitions were specifically developed for bleeding occurring after CABG [10]. The clinical significance of most definitions has been evaluated and validated to date only by their proposers [11]. The aim of the present study was to validate and compare the prognostic value of different bleeding definitions in patients undergoing off-pump coronary artery bypass grafting (OPCAB).

## Methods

### Patient population and data collection

Our retrospective, single-center, cohort study enrolled a total of 3988 consecutive patients aged > 18 years who had undergone isolated OPCAB between February 2008 to December 2014 in Beijing Anzhen Hospital (Beijing, China), including emergency and elective operations performed in off-pump setting. The major exclusion criteria were: 1) preoperative exposure to oral anticoagulants including warfarin and direct oral anticoagulants, 2) preoperative severe renal insufficient, 3) undergoing any other major cardiac surgery procedure including valvular repair or replacement, 4) and with insufficient records to specify bleeding events. The detailed study flowchart is depicted in Fig. 1. All patients provided written informed consent for the procedure and subsequent clinical data for retrospective analysis on the day of admission. The ethical review and informed consent of this study were approved by institutional ethics committee of Beijing Anzhen Hospital, Capital Medical University. The protocols of our study obeyed the principles of the 1983 Declaration of Helsinki.

**Fig. 1:** Study flowchart

All data used int the present study was collected from the electronic medical records by two trained medical staffs. The important data information was monitored and revised by a third medical staff to ensure the accuracy. The database of the electronic medical system contained the baseline and operative data and immediate postoperative adverse events, which provided available complete pre-, intra-, and postoperative data for all included patients.

### Endpoints and definitions

The primary endpoint of this study was a composite of in-hospital death and postoperative myocardial infarction (MI). In-hospital death included all-cause death before discharge and post operation. The postoperative MI was defined as nonfatal elevation of cardiac troponin (cTn) values > 10 times the 99th percentile upper reference limit (URL) in patients with normal baseline cTn values [12]. The secondary endpoint was postoperative acute kidney injury (AKI) which was defined as an acute postoperative renal insufficiency resulting in one or more of the following in the first 48 h after surgery as proposed by Acute Kidney Injury Network (AKIN) as stage 1 of acute kidney injury: 1) an increase of serum creatinine level of ≥0.3 mg/dl (≥ 26.4 μmol/l); 2) at least a 50% greater increase in creatinine above baseline preoperative level (1.5-fold from baseline); 3) a reduction in urine output (documented oliguria of less than 0.5 ml/kg per hour for more than six hours) [13].

Major bleeding events were assessed and adjudicated according to the classification from European registry of Coronary Artery Bypass Grafting (E-CABG), [8] the Universal Definition of Perioperative Bleeding (UDPB), [9] the Bleeding Academic Research Consortium (BARC) [14] classification and the classification from Study of Platelet Inhibition and Patient Outcomes (PLATO) [15].

### Statistical analysis

Baseline continuous variables were presented as mean value ± standard deviation if normally distributed and otherwise as median (interquartile range). Categorical variables are expressed as percentages.

Multivariable logistic regression analysis was used to investigate the association between perioperative major bleeding and endpoints adjusting for potential confounding factors which had been reported in previous studies, using forward stepwise selection to identify significant confounding variables. Potential confounders reported in previous studies as important determinants of perioperative outcomes and variables suggested to be associated with clinical outcomes by univariate logistic analysis would be offered to the logistic regression models. Power of the association between risk factors and outcomes was expressed as odds ratio (OR) and 95% confidence intervals (CI). Goodness-of-fit tests of − 2 log likelihood were used to evaluate the improved model performance comparing models with and without bleeding.

Statistical analysis was performed with the SPSS version 24.0 statistical software (IBM Corporation, Armonk, New York, USA). All statistical tests were 2-sided and results were considered to be statistically significant at a *p* value < 0.05.

## Results

Baseline demographic characteristics of the overall 3988 patients included in the present study were reported in Table 1.

**Table 1:** Baseline Characteristics

Variable	No. (%) / Mean + SD
Age (years)	62.15 ± 9.10
Female gender	947 (23.75%)
BMI (kg/m2)	25.72 ± 3.18
SBP (mmHg)	129.07 ± 19.19
LVEF (%)	56.11 ± 10.04
LVEF< 40%	119 (2.98%)
Hemoglobin (g/L)	139.25 ± 16.23
BMI ≤ 25	1764 (44.23%)
Hypertension	2600 (65.20%)
Diabetes	1411 (35.38%)
Hyperlipidemia	922 (23.12%)
Prior MI	566 (14.19%)

### Bleeding events and clinical outcomes

In the 3988 OPCAB patients analyzed, in-hospital mortality was 1.23% (*n* = 49) and postoperative MI occurred in 5.01% (*n* = 200) of patients. And 24.70% (*n* = 985) of patients suffered from AKI after procedure.

BARC CABG-related bleeding (type 4) occurred in 168 (4.21%) patients. The incidence of major bleeding defined by E-CABG class 2–3 and UDPB class 3–4 were 4.16% (*n* = 166) and 9.85% (*n* = 393). And the incidence of major bleeding according to PLATO criteria was 36.28% (*n* = 1447). All major bleeding events defined as E-CABG class 2–3 were concomitantly captured in both BARC type 4 and UDPB class 3–4 bleeding (98.8% in BARC type 4 and 42.2% in UDPB class 3–4). The incidence rates of adverse outcomes including composite endpoints, in-hospital death, MI and AKI among patients with minor or major bleeding classified by different bleeding classifications were summarized in Table 2. Among patients with bleeding events, increasing grades of E-CABG and UDPB classifications but not PLATO were associated with increasing risk of in-hospital death (*p* < 0.001).

**Table 2:** Incidence of adverse events after procedure according to various bleeding classification

Classifications/Outcomes	Severity of perioperative bleeding				
UDPB	0	1	2	3	4
Composite outcomes [n (%)]	118 (6.37%)	21 (5.36%)	70 (5.18%)	24 (8.22%)	19 (18.81%)
In-hospital death [n (%)]	18 (0.97%)	2 (0.51%)	16 (1.18%)	4 (1.37%)	9 (8.91%)
MI [n (%)]	99 (5.35%)	17 (4.34%)	53 (3.92%)	18 (6.16%)	13 (12.87%)
AKI [n (%)]	375 (20.25%)	82 (20.92%)	400 (29.61%)	85 (29.11%)	43 (42.57%)
BARC	without Type 4	Type 4: CABG-related bleeding			
Composite outcomes [n (%)]	229 (5.99%)			23 (13.69%)	
In-hospital death [n (%)]	40 (1.05%)			9 (5.36%)	
MI [n (%)]	183 (4.79%)			17 (10.12%)	
AKI [n (%)]	919 (24.06%)			66 (39.29%)	
PLATO	minimal bleeding	minor bleeding	other major bleeding	major life-threatening bleeding	
Composite outcomes	35 (6.22%)	1 (5.88%)	89 (4.74%)	114 (7.45%)	
In-hospital death	4 (0.71%)	0	12 (0.64%)	33 (2.16%)	
MI	32 (5.68%)	1 (5.88%)	78 (4.15%)	89 (5.82%)	
AKI	121 (21.49%)	5 (29.41%)	422 (22.47%)	437 (28.56%)	
E-CABG	0	1	2	3	
Composite outcomes	147 (5.94%)	69 (5.13%)	20 (12.42%)	3 (42.85%)	
In-hospital death	23 (0.97%)	17 (1.26%)	6 (3.73%)	3 (42.85%)	
MI	128 (5.17%)	55 (4.09%)	12 (7.45%)	2 (28.57%)	
AKI	506 (20.44%)	413 (30.71%)	60 (3.79%)	6 (85.71%)	

### Multivariable logistic model and comparison of classifications

The results of the multivariable logistic models to evaluate the association between bleeding and adverse outcomes were shown in Table 3. BARC type 4 bleeding which was specific for bleeding related to CABG was independently associated with a more than 2-fold increase in risk of in-hospital death and postoperative MI (OR = 2.54, 95% CI: 1.66–4.19, *P* < 0.001). Major bleedings defined as E-CABG class 2 and 3 (class 2: OR = 2.24, 95% CI: 1.36–3.70, *P* = 0.001; class 3: OR = 12.65, 95% CI: 2.74–18.43, *P* = 0.002) or UDPB class 4 (OR = 3.52, 95% CI: 2.05–6.02, P < 0.001) were significantly associated with poorer perioperative clinical outcomes.

**Table 3:** Association of bleeding and primary endpoints according to multivariable models

	OR	95% CI		*p*-value
		Lower	Upper	
BARC type 4 bleeding	2.64	1.66	4.19	< 0.001
E-CABG				
1	0.87	0.65	1.17	0.363
2	2.24	1.36	3.70	0.002
3	12.65	2.74	58.44	0.001
UDPB				
1	0.78	0.47	1.28	0.319
2	0.80	0.59	1.10	0.172
3	1.25	0.77	2.02	0.365
4	3.52	2.05	6.02	< 0.001
PLATO				
Minor	0.89	0.11	6.97	0.910
Other major	0.75	0.49	1.13	0.162
Major life-threatening bleeding	1.19	0.79	1.80	0.398

We created a multivariable model using baseline characteristics such as age, gender, BMI, diabetes, hypertension, prior MI, renal insufficiency, decreased left ventricular ejection fraction (LVEF), systolic blood pressure (SBP) values and preoperative haematocrit (Hct) values and different bleeding classifications were added to this multivariable model to evaluate whether the inclusion of bleeding events could improve the predictive value of this model. The inclusion of bleeding stratified by BARC, E-CABG and UDPB improved the prediction of in-hospital death and postoperative MI (Table 4). BARC type 4 bleeding and E-CABG class 2–3 bleeding improved the model to similar degrees.

**Table 4:** Improvement in predictive value of multivariable model

	Change in -2log likelihood vs. Baseline Model	*p*-value
Baseline + BARC type 4	1794.27–1780.49 = 13.78	< 0.001
Baseline + E-CABG class 2–3	1794.27–1780.50 = 13.77	< 0.001
Baseline + PLATO major	1794.27–1788.79 = 5.48	0.222
Baseline + UDPB class 3–4	1794.27–1781.79 = 12.48	< 0.001

## Discussion

Our results indicated that BARC, E-CABG and UDPB but not PLATO classifications can effectively stratify the severity of postoperative bleeding. Moreover, bleedings classified as BARC type 4, E-CABG class 2 and 3 and UDPB class 4 were independently associated with an increased risk of in-hospital death and postoperative MI.

Bleeding has been recognized as important determinants of outcomes after cardiac surgery according previous studies [16–18]. Quantifying the amounts of blood products transfusions is an important factor to measure the severity of bleeding. A study from Koch et al. demonstrated the correlation between RBC transfusion and increased risk of postoperative morbid events including mortality, renal failure, prolonged ventilatory support, serious infection, cardiac complications and neurologic events, along with increased costs of care [19, 20]. Even minor transfusion such as 1 and 2 units of red blood cells is significantly associated with increased morbidity and mortality after OPCAB [21]. Reexploration for bleeding is also a common factor in different bleeding classification, which has been reported to be an important source of morbidity after cardiac surgery [22]. Therefore, an effective stratifying system for bleeding events according to bleeding-related factors is helpful and necessary to estimate outcomes of cardiac surgery. Although several stratifying systems for severity of perioperative bleeding have been proposed, validation on their prognostic significance was required.

In accordance with our results, the UDPD classification was suggested to have an important effect on both short- and long-term survival after CABG by several studies [7, 23]. Kinnunen et al. evaluated the clinical significance of UDPB classification in patients undergoing isolated CABG and observed the association between high UDPB classes and poorer immediate and late outcomes [23]. In addition to mortality, other adverse outcomes including AKI and low cardiac output were also associated high UDPB classes bleeding. In our recent study, we have confirmed that perioperative bleeding defined as the UDPB class 3 to 4 bleeding was associated with a higher risk of postoperative AKI in ACS patients who underwent OPCAB [24]. The UDPB classification was based on the amount of chest tube blood loss, use of blood products and the need of reexploration or delayed sternal closure. Nevertheless, the need of data on transfusion of 6 different blood products makes its application complicated and limited its use in clinical and research activities.

BARC type 4 bleeding is the only one specific CABG-related bleeding definition [14]. Bleeding events are much more common in CABG. And transfusion is inherent to cardiopulmonary bypass which makes it difficult to define a threshold for bleeding in CABG [25]. Therefore, it is necessary to definite CABG-related, and non–CABG-related bleeding separately. BARC type 4 bleeding used the same criteria as the bleeding in the setting of CABG defined by the Thrombolysis in Myocardial Infarction (TIMI) [2, 26] bleeding definition which integrated mainly laboratory-based data. It has been confirmed to be associated with 4 to 5 times higher risk of mortality [10]. The E-CABG classification measures the severity of bleeding by quantifying the amount of blood products administered to correct anemia and prevent further blood loss as well as reexploration for bleeding. The E-CABG bleeding has been shown robust association with adverse events, such as in-hospital death and prolonged intensive care unit stay, after cardiac surgery [8, 27]. On the contrary, the PLATO classification in which drop of hemoglobin played an important role showed poor predictive performance of clinical likely because it was poorly applicable to surgical patients. And BARC classification type 1 to 3 were excluded due to its similarity with PLATO [28]. It is noteworthy that decrease in hemoglobin or hematocrit is always included in bleeding definition for nonsurgical operation, such as PLATO bleeding and TIMI non-CABG related bleeding, rather than bleeding definition for surgical operation which emphasize the intervention to reduce ongoing bleeding including blood products transfusion.

The present study provided validation of four different bleeding classification in a large cohort of patients undergoing CABG. We observed that bleeding defined as BARC type 4, E-CABG class 2 and 3 and UDPB class 4 carried a higher risk of in-hospital death and postoperative MI as well as AKI. Such results of our study confirmed that BARC, E-CABG and UDPB were promising research tools for stratification of bleeding risk. Appropriate stratification of bleeding events can provide prognostic information and be useful for estimating the risk of adverse outcomes.

There are some limitations in our study that must be acknowledged. Firstly, the retrospective nature of the present study was an important limitation and prospective data collection might yielded better source documentation to classify bleeding complication. However, the data regarding hemoglobin, transfused blood products and outcomes in hospital were retrieved from medical records system which was considerably reliable. Secondly, the lack of data on follow-up after surgery prevented us to evaluate the long-term effect of major bleeding on the clinical outcomes. But majority of bleeding events and adverse events resulting from bleeding occurred during perioperative period. Thirdly, the present study only enrolled patients undergoing OPCABG and further studies are needed to investigate the prognostic significance of bleeding classifications in patients undergoing other cardiac surgery.

## Conclusions

Our present study confirmed that bleeding assessed by BARC, E-CABG and UDPB classifications were significantly associated with poorer immediate outcomes but not PLATO classifications. These classifications seemed to be valuable tool in the assessment of prognostic effect of perioperative bleeding events on clinical outcomes. And the significance of these bleeding classifications needs to be validated in a larger population undergoing other cardiac surgery.

## Data Availability

The data and other material of this study were available by contacting the corresponding authors.

## Abbreviations

AKI: Acute kidney injury
BARC: Bleeding academic research consortium
CABG: Coronary artery bypass grafting
E-CABG: European registry of coronary artery bypass grafting
MI: Myocardial infarction
OPCAB: Off-pump coronary artery bypass grafting
PLATO: Platelet inhibition and patient outcomes
UDPB: Universal definition of perioperative bleeding
URL: Upper reference limit
